The article "Teaching of Dance Choreography Course Based on Multimedia Network Environment" was retracted in 2023. Reasons: unreliable results or conclusions; concerns about the data; concerns about the peer review; concerns about the citations.

# Teaching of Dance Choreography Course Based on Multimedia Network Environment

**DOI:** 10.1155/2022/8627822

**Published:** 2022-09-10

**Authors:** Yue Sun

**Affiliations:** Department of Dance, School of Music and Dance, Harbin University, Harbin 150028, China

## Abstract

The growth of society has been significantly impacted by the introduction of the new multimedia era. A new task will present itself to the choreographer in light of this context. This paper makes the argument that multimedia technology should be incorporated with dance art so that dance works can give audiences a deeper feeling and impression and promote the diversified development of dance art by outlining the characteristics of multimedia and its application advantages in choreography. A multimedia network classroom contains a variety of features, including real-time educational feedback, an interactive learning environment, and a diverse instructional content. Based on this, this article builds and integrates the instructional resources for the dance choreography course as well as the instructional management system for the course. In order to precisely and effectively teach choreography, it is necessary to give the proper instructional materials. According to experimental findings, the recall and precision of the suggested method can both approach 95.71% and 96.84%, respectively. It partially resolves the issues of users having trouble locating necessary educational resources and instructional resources being underutilised. The dance choreography course is being taught using this way in a multimedia network setting.

## 1. Introduction

Multimedia is a byproduct of modern society and is present in all facets of life, including the dissemination of information and the widespread use of network technology. With the advancement of contemporary information technology, multimedia education has emerged as a novel instructional method [1]. Due to its features of digitalization, multimedia, vast information, intense engagement, and extensive coverage, it overcomes the time and space constraints of traditional teaching and offers opportunities for more individuals to obtain education. Dance is a classic art form that is currently popular in the age of multimedia. It is a once-in-a-lifetime chance as well as an unexpected challenge for dance [2]. At present, people's appreciation of art has more diverse perspectives, and the sense of science and technology and futurity have become new elements in dance creation. Dance choreography teaching is mainly to teach dance-related knowledge and skills through teachers, so as to encourage students to continuously acquire corresponding dance knowledge. This instructional course is an activity of mutual influence and interaction between teachers and students [3]. To cultivate professional choreographers, we should not only teach their dance skills but also enrich their professional theoretical knowledge and music appreciation ability. As an excellent dancer, one should not only master exquisite dance skills but also have a high artistic accomplishment [4]. It can be said that dancers' artistic feeling of dance is their understanding of music and their understanding of dance. As a dance art that expresses thoughts, feelings, and plots through dance movements, in the process of creating dance works, multimedia technology makes all aspects of choreography form a unified organic whole, which is of great significance.

The article "Teaching of Dance Choreography Course Based on Multimedia Network Environment" was retracted in 2023. Reasons: unreliable results or conclusions; concerns about the data; concerns about the peer review; concerns about the citations.

Under the influence of multimedia background, the creation and dissemination of art gradually attached to multimedia and began a profound evolution [5]. On the one hand, multimedia promotes the circulation of art, which makes the originally relatively small art categories push to the mass market; on the other hand, the expanding market and audience also play an important role in influencing artistic creation. The application of multimedia instructional means to the dance choreography instructional course can effectively promote the smooth progress of instructional activities and make the relevant dance knowledge and skills be displayed to students in a vivid and lively form [6]. At the same time, it can bring new vitality to modern dance creation and help to shape dance image, organize dance language, design dance segment arrangement, and other links better. Using multimedia network environment to teach dance choreography course is of great significance to stimulate students' learning interest, enhance students' learning ability, and improve the overall teaching quality [7]. Multimedia teaching management is a practise in which managers adhere to the principles of teaching, make decisions and organise instructional activities, logically allocate and use instructional resources, adopt multimedia technology, take students into consideration, and use other management techniques and modern educational theories [8]. This is done in order to achieve the best teaching goals in the computer network environment. Similar to how other disciplines are integrated, the effective integration of multimedia technology and dance course instruction must be guided by advanced teaching theory. Without the direction of advanced theory, practise is blind, and successful integration is impossible. The specific use of multimedia instructional techniques in the teaching of choreography is the topic of this essay, which also analyses and discusses this application in an effort to identify the benefits of using multimedia instructional methods in the teaching of choreography. This article produces and integrates the instructional resources for the dance choreography course and builds the instructional management system for the course on the basis of the information presented. These are the primary innovations of this study:

1. By expounding the characteristics of multimedia and its application advantages in choreography, this paper puts forward that multimedia technology should be integrated with dance art, so that dance works can give audiences a deeper feeling and impression and promote the diversified development of dance art. At the same time, it is suggested that the multimedia network classroom should make use of the diversity of instructional information, the interactivity of instructional system, the real-time instructional feedback, and many other characteristics to make a new attempt in the teaching of dance choreography
2. In this paper, the instructional management system of dance choreography course is constructed, and a feasible scheme of developing and integrating instructional resources of dance choreography course is designed and implemented. At the same time, an improved flow scheduling algorithm and cache replacement strategy are proposed. In this paper, information integration in instructional resources is realized by extracting ontology from relational database and integrating ontology, which is beneficial to increase new resources and reuse existing ontology. It solves the problems that multiontology method is difficult to add new sources, and hybrid method is difficult to reuse existing ontology. It improves the individuation and intelligence of the instructional management system of dance choreography course

The article "Teaching of Dance Choreography Course Based on Multimedia Network Environment" was retracted in 2023. Reasons: unreliable results or conclusions; concerns about the data; concerns about the peer review; concerns about the citations.

## 2. Related Work

Zhang pointed out that the information-based classroom should get rid of the “teacher-centered” way of thinking, actively exert students' participation, and improve students' innovative ability [9]. In the instructional process, teachers should try their best to give students enough space for interaction and communication, so as to truly realize the unity of dominance and subject. Ali et al. believe that multimedia technology is a computer technology that comprehensively processes image, text, sound, and video information and makes it integrated and interactive [10]. Yang et al. noted that multimedia technology is outfitted with information elements like images, texts, and sound animations, which may simultaneously provide users with rich sensory experiences and deliver information from a variety of angles [11]. The idea of loose and organised management of instructional resources was put forth by Gomez et al. [12], which protects the complexity and diversity of instructional resources. According to Guan et al., the integration of teaching and information technology offers a good platform for instruction and enhances the curriculum, while also piquing students' interest in the subject and enhancing the effectiveness and calibre of classroom instruction [13]. According to Monique and Malini, cutting-edge teaching techniques can improve the depth of dance education courses, making them simpler to comprehend and accept [14]. Pastore and Pentassuglia systematically analyzed the technical basis, network teaching characteristics, and network teaching management of the multimedia network teaching management platform [15]. And it is on this foundation that the core ideas behind multimedia network teaching management are developed. According to Ke's research, the Web has multiple communication channels that can facilitate in-depth discussions between teachers and students as well as among students, making it an effective teaching tool that can be used from anywhere and at any time [16]. This is crucial for raising teaching standards and encouraging the growth of pupils' highly developed cognitive abilities. According to Haskell, modern teaching should actively respond to the needs of the society for development and grasp the orientation of talent cultivation, pay more attention to the development of innovation ability, maximise the talents of learners, and mobilise their zeal and initiative in order to ultimately cultivate high-quality talents [17]. Qi et al. made some useful explorations and attempts on the open instructional mode based on the multimedia network by using the existing multimedia network environment in schools [18]. Qiao pointed out that the load balancing of servers is the basic guarantee for reliable and efficient data access, especially the research on the balancing of instructional resource servers with high load is particularly important [19].

This paper makes the argument that multimedia technology should be incorporated with dance art so that dance works can give audiences a deeper feeling and impression and promote the diversified development of dance art by outlining the characteristics of multimedia and its application advantages in choreography. Based on this, this article develops a practical plan for the development and integration of instructional resources for a dance choreography course as well as the instructional management system for the course. A better flow scheduling technique and a cache replacement strategy are both suggested at the same time. The study demonstrates that this approach enhances the personalisation and intelligence of the dance choreography course's instructional management system and to some part resolves the issues of users' difficulties in locating necessary instructional resources and low rate of resource usage.

The article "Teaching of Dance Choreography Course Based on Multimedia Network Environment" was retracted in 2023. Reasons: unreliable results or conclusions; concerns about the data; concerns about the peer review; concerns about the citations.

## 3. Methodology

### 3.1. Multimedia Dance Choreography Teaching

Multimedia's emergence and progress are inextricably linked to the advancement of electronic equipment like computers and network technologies, which gives multimedia development a more fresh feel. Additionally, technology's openness allows for more freedom in the creation of multimedia, which has drastically altered people's lives [20]. Multimedia network technology is currently employed extensively in the educational sector. In addition to traditional teaching, correspondence teaching, and network teaching, lifelong education and lifetime learning will increasingly rely on online teaching, electronic distance learning, virtual teaching, and network teaching. A variety of media are logically integrated through the use of multimedia technology, which integrates information in the form of text, graphics, images, animation, video, and audio into a real-time and interactive systematic presentation of information. Multimedia instructional means mainly refer to the effective design and management of instructional resources and instructional process through the effective application of various multimedia technologies such as computers, so as to optimize teaching objectives and enhance the flexibility of instructional courses. At present, multimedia is based on digital technology, using computer language as the main body, transforming the media form into digital form, so that it can exist as hypertext [21]. It also features network and virtual characteristics due to its reliance on network speed, and interactivity can be improved by multimedia. Teachers assume the roles of organiser, instructor, helper, and promoter during the entire educational process in open teaching that is based on multimedia. In order for students to effectively create the meaning of what they have learned at this time, teachers should make full use of the learning environment aspects such as circumstance, cooperation, and dialogue as well as students' initiative, enthusiasm, and innovative spirit. The following are some features and benefits of multimedia technology:

(1) *Interactivity*. Interactivity means that users can interact with various information media of computers, thus providing users with more effective means to control and use information

(2) *Complexity*. Complexity mainly refers to the diversification of information processing means of multimedia technology, which can also be called the diversification or multidimension of media. It breaks the limitation of the original simplification of data and information

(3) *Integration*. All kinds of information, materials, and software equipment of multimedia technology need to be integrated

As a traditional art form, dance is in the wave of multimedia era. For dance, it is not only an unprecedented opportunity but also a sudden challenge. Dance is an art that expresses people's emotions and deduces the content and plot of a story with human movements, gestures, and expressions. It can be said that dance itself is the most direct, vivid, and infectious in expressing people's thoughts and feelings. In order to gradually increase student comprehension and acceptance during the dance teaching process and help students learn important knowledge and skills more efficiently, instructional approaches must be constantly improved. The teaching of dance choreography using multimedia technology respects the laws of educational development and the development of multimedia technology, focuses on changing teachers' concepts, pushes teachers to adopt contemporary educational concepts, and accomplishes teaching goals through the use of multimedia courseware and collaboration between various instructional methods. It's challenging to put into words the particular connotation of dance, which makes teaching choreography challenging. The instructor's live presentation is typically the most intuitive method. The use of multimedia helps compensate for the shortcomings of conventional choreography instruction. Through the use of multimedia technology, the style and content of dance may be graphically shown and regularly viewed, in part assisting students in expanding their knowledge and comprehension of the choreographer. It is a reciprocal process, absorbing the student-centered instructional design idea, allowing students to explore, think, and discover independently, allowing every student to experience the process of knowledge discovery or “creation” from time to time, and inspiring students' creative enthusiasm. Choreography is a special art, which requires special instructional methods and means [22]. The introduction of multimedia has greatly altered how choreographers shape dance imagery, organise dance vocabulary, arrange design, and organise dance instruction. The emergence of multimedia can modernise traditional choreography by adding fresh elements and making full use of multimedia resources. In order to deliver a high-quality education, we should actively promote the use of multimedia information technology in dance teaching, adopt a variety of instructional methods, and create a vibrant learning environment. The choreographer can use the information integration and management of multimedia to deliberately choose the material taught on stage, take into account how the forms on and off the stage complement one another, and arouse enthusiasm on both sides attaining the goal of emphasising important information and increasing effectiveness.

The article "Teaching of Dance Choreography Course Based on Multimedia Network Environment" was retracted in 2023. Reasons: unreliable results or conclusions; concerns about the data; concerns about the peer review; concerns about the citations.

### 3.2. Dance Choreography and Creation from the Perspective of Multimedia

The diversity of dance lies not only in its forms of expression, stage art, and creative techniques but also in its rich cultural background. With the emergence of multimedia, dance creation can be combined with multimedia, and creative means can be more diversified. Teachers can store videos and pictures related to dance teaching into related multimedia devices before the course teaching. By playing them to students in the classroom, students can capture some effective related information during their own viewing, thus continuously enhancing students' understanding and learning ability. Multimedia technology is like a demonstrator who does not know fatigue. It can repeat the same action endlessly and accurately, so that students can try to figure out the elements of the action repeatedly until they master and truly appreciate the essence and essence of the dance action. In addition, the creation of the environmental atmosphere of dance works is a bonus of creation. In the construction of environmental atmosphere, the use of video broadcasting can have a positive impact on the information transmission of dance works and the creation of vivid atmosphere. Multimedia technology can also be used to build futuristic dance pieces and add high-tech components to existing dance works. The entire demonstration is a significant use of multimedia technology that demonstrates to pupils the entire training combination or continuous action combination that must be taught in a stage thoroughly and systematically. Students can greatly improve their understanding of dance movements under the direction of the comprehensive and methodical demonstration teaching method, allowing them to successfully integrate some particular dance movements, which is crucial to the study of this course in dance choreography. By doing this, teachers can present to students in an intuitive way the crucial and challenging elements of their actions as well as the challenges they face when instructing and improving the effectiveness and quality of their instruction.

When a choreographer creates a dance, the material selection can be real events, literary works, historical events, myths and legends, etc. As one of the artistic sources of these choreographers, with the help of multimedia technology, the situation at that time can be restored as much as possible, or the imagination can be fully explained. Driven by thinking, dance choreographers will be able to innovate their own thinking concepts and present a more real side of dance. This can make the audience fully integrate into the scene and feel the artistic charm and value of dance. In addition, in order to enhance the public's attention to art, apart from creating infectious works, it is also necessary for the public to have wider access to works and experience the aesthetic feeling of art. The application of projection equipment and VR technology can not only create a stage atmosphere but also put pictures into the audience area, create an artistic atmosphere in the audience's environment, and stimulate the audience's enthusiasm for participation, thus presenting interactive performances. In the teaching of modern dance choreographer, using information network technology can create a multimedia demonstration environment, which can make people intuitively feel and appreciate the artistic charm of dance. The application of modern technology in situational teaching can fully tap and exert students' imagination and creativity and realize the effect of digital aesthetic education. Nowadays, there are more and more kinds of dances, such as modern dance, contemporary dance, and modern ballet. However, the existing dance appreciation textbooks only mention some old works, and the teaching content of teachers cannot keep up with the modern development and changes. Therefore, it is necessary to build an instructional resource database of dance choreography course. Through the establishment of dance information resource database, students can occupy the image resources of dance to a greater extent and expand their learning horizons and fields. At the same time, it also saves the resources of dance teaching to a certain extent.

The article "Teaching of Dance Choreography Course Based on Multimedia Network Environment" was retracted in 2023. Reasons: unreliable results or conclusions; concerns about the data; concerns about the peer review; concerns about the citations.

### 3.3. Construction of Instructional Management System of Choreography Course

The grid will realise the connectivity of all Internet resources, just as the traditional Internet already realises the connection of computer hardware, the Web already realises the connection of web pages. Grid technology allows for the Internet to be expanded into a sizable processing and service platform, improving the management of online resources. In a dynamically changing network environment, it may share resources and work out issues cooperatively, giving users access to flexible, intelligent, and cooperative information services as well as a level of ease and power never before possible. This work uses metadata to refer to knowledge points as atomic resources in order to conceal the diversity and differences of knowledge points in various courses. The logical and structural laws among atomic resources, however, are governed by the principles of human learning and cognition. Therefore, a single paradigm for structured combination and management is adopted in this research. In this approach, educational resources also fit the definition of grid resources and can be used to manage and manipulate grid resources. Information integration is to make it possible for heterogeneous data sources to share information, make better use of available resources, and enhance overall system performance. Integrating information should therefore accomplish two objectives: distribution transparency and heterogeneous data source transparency. The instructional management system of dance choreography course in this paper is a B/S architecture system. PC users and mobile phone users can access the system through the network and interact with the server. The architecture diagram of instructional management system of choreography course is shown in Figure 1.

In the multimedia on-demand system, users have a strong tendency to access multimedia files, and this tendency directly affects the performance of the whole system. In this paper, block access frequency and user's stopping access probability are used as the criteria for quantitative analysis of internal access tendency. An evaluation vector can be established with all instructional resources of users.

(1) $$\begin{array}{c} E_{i}=\left(x_{1},x_{2},x_{3},\cdots ,x_{j}\right), \end{array}$$

where *x*_*j*_ is the rating made by the user to the resource, which can be the original rating value or the quantized value. The data source layer of this paper selects relational database as the provider of system data, which is a preexisting, heterogeneous, and autonomous data source in the integrated environment. In the process of extracting ontology from relational database, we use knowledge base to supplement the extracted ontology and strive to make the extracted ontology completely consistent. The preprocessing of system load data is mainly to preprocess the abstract time series to meet the input requirements of time series analysis model.

Assuming that the system can provide concurrent access to *N* users at the same time, the duration of the video program in the server is *T*. The user's video on demand obeys the Poisson distribution *λ*(*n*), then the average number of requests within the *t* duration is *λ*∗*t*, and the rejection rate of the video server is

(2) $$\begin{array}{c} \rho =\text{Rejected quantity}/\text{Total visits}=1-N/\left(1+\lambda T\right). \end{array}$$

Therefore, if the video file is divided, the service response rate of the server can be improved, but at the same time, the request frequency of users to the server will be increased. Determine whether {*x*_*t*_} is a nonstationary time series and contains trend items. If so, first extract the trend item *d*_*t*_ contained in {*x*_*t*_}.

(3) $$\begin{array}{c} y_{t}=x_{t}-d_{t}. \end{array}$$

From this, the stationary time series {*y*_*t*_} can be obtained, and the time series can be modeled accordingly. For the trend term {*d*_*t*_}, multiple regression and other methods can be used to estimate from the time series {*x*_*t*_}, and then *y*_*t*_ and *d*_*t*_ are combined to calculate the final model. When the time series {*x*_*t*_} is a stationary time series and the mean value is not equal to zero, the mean value ${\hat{\mu }}_{x}$ of the series needs to be calculated, and it is zeroed according to the following formula to obtain a new series {*y*_*t*_} for modeling. The time series that modeling can be applied to are all zeroed time series, as follows:

(4) $$\begin{array}{c} y_{t}=x_{t}-{\hat{\mu }}_{x}. \end{array}$$

In the cosine similarity method, it is assumed that the scoring information of user *i* and user *j* in the *n* dimension resource entry space is represented as vectors $\bar{S_{i}}$ and $\bar{S_{j}}$, respectively, then the similarity Sim(*i*, *j*) between them can be defined as

(5) $$\begin{array}{c} \text{Sim}\left(i,j\right)=\cos\left(\bar{S_{i}},\bar{S_{j}}\right)=\frac{\bar{S_{i}}\times \bar{S_{j}}}{\left\|\bar{S_{i}}\right\|\times \left\|\bar{S_{j}}\right\|}. \end{array}$$

In the related similarity measurement method, assuming that the set of resource items scored by user *i* and user *j* is represented by *I*_*i*,*j*_ = *I*_*i*_∩*I*_*j*_, the similarity Sim(*i*, *j*) between them can be defined as

(6) $$\begin{array}{c} \text{Sim}\left(i,j\right)=\frac{\sum_{x\in I_{i,j}}\left(r_{jx}-{\bar{r}}_{j}\right)\left(r_{ix}-{\bar{r}}_{i}\right)}{\sqrt{\sum_{x\in I_{i,j}}{\left(r_{jx}-{\bar{r}}_{j}\right)}^{2}}\sqrt{\sum_{x\in I_{i,j}}{\left(r_{ix}-{\bar{r}}_{i}\right)}^{2}}}, \end{array}$$

where *r*_*ix*_ represents the rating of resource item *x* by user *i*; *r*_*jx*_ represents the rating of resource item *x* by user *j*; ${\bar{r}}_{i}$ and ${\bar{r}}_{j}$ represent the average item rating of user *i* and user *j*, respectively. Assuming that the nearest neighbor user set of user *x* can be expressed as *U*, the predicted score *P*_*x*,*i*_ of the target user for resource item *i* can be calculated by the following formula:

(7) $$\begin{array}{c} P_{x,i}=\bar{S_{x}}+\frac{\sum_{y\in U}\left(\text{Sim}\left(x,y\right)\times \left(S_{y,i}-\bar{S_{y}}\right)\right)}{\sum_{y\in U}\left(\text{Sim}\left(x,y\right)\right)}. \end{array}$$

Among them, Sim(*x*, *y*) represents the similarity measure of user *x* and user *y*; *S*_*y*,*i*_ represents the score of resource item *i* by user *y*; $\bar{S_{x}}$ and $\bar{S_{y}}$ represent the average resource score of user *x* and user *y*, respectively.

The article "Teaching of Dance Choreography Course Based on Multimedia Network Environment" was retracted in 2023. Reasons: unreliable results or conclusions; concerns about the data; concerns about the peer review; concerns about the citations.

This study uses the average value of attribute similarity as a proxy for the final conceptual attributes when calculating the similarity of conceptual attributes. The maximum values are removed, respectively, for each row and column of the similar matrix, and the sum is then obtained by adding them. Record as

(8) $$\begin{array}{c} \text{MaxSumSim}\left(X_{1},X_{2}\right). \end{array}$$

The similarity of concepts is recorded as follows:

(9) $$\begin{array}{c} \text{Arrsim}\left(X_{1},X_{2}\right). \end{array}$$

Therefore, the similarity calculation formula of conceptual attributes is as follows:

(10) $$\begin{array}{c} \text{Arrsim}\left(X_{1},X_{2}\right)=\frac{\text{MaxSumSim}\left(X_{1},X_{2}\right)}{\text{Size}\left(X_{1}\right)+\text{Size}\left(X_{2}\right)}. \end{array}$$

Calculate the average similarity between conceptual attributes by dividing the highest similarity between each attribute and other characteristics by the total number of attributes. Further processing is done on the calculation results, so the range of similarity is [0, 1]. The following is the normalisation formula that is suggested in this paper:

(11) $$\begin{array}{c} \text{Sim}\left(x,y\right)=1-{u_{0}}^{\text{Sim}\left(x,y\right)} \end{array}$$

In the formula, *u*_0_ is the normalization factor, which is a positive real number greater than 1. It can be seen from the change curve of the value of the function, when the value of *u*_0_ is larger, the speed of the calculation result approaching 1 is faster.

The video server must be able to deliver a large number of concurrent access services in order to handle the demand for media videos from numerous users. The processing power and I/O capacity of servers are starting to act as a bottleneck in the delivery of services due to the rising demand for video. This paper adopts multiple servers to accommodate the demands of numerous concurrent accesses due to the inherent performance limitations of a single server. The system administrator is in charge of managing educational resources and setting up various system applications, while teachers and students use the system and benefit from the application services it offers. Users' interactive data of all types will be uniformly stored in the system database. The structure diagram of choreographer course instructional management system is shown in Figure 2.

The article "Teaching of Dance Choreography Course Based on Multimedia Network Environment" was retracted in 2023. Reasons: unreliable results or conclusions; concerns about the data; concerns about the peer review; concerns about the citations.

The purpose of information integration is to establish a unified access interface on the logical layer of data sources and realize distributed sharing of heterogeneous data sources. At this point, the global query that we can provide to users can be completed directly on the integrated global ontology, and then the results are returned to users. This is the main application of information integration in this paper, and users can easily realize global query. The typical characteristics of real-time data streams such as online video, audio, and images are that their storage consumption is potentially unbounded; its statistical characteristics, such as generation order and interval, are uncertain. Therefore, the real-time data stream consumes a lot of resources of the resource server, which easily leads to the paralysis of the server and is also the main factor leading to the unbalanced load of each server. In view of the network congestion caused by video communication and the serious load brought to the video server, an effective method is to use proxy server, that is, to achieve this goal by caching some or all data needed by most users in the proxy server. In addition, the user information base, instructional resource base, and user behavior information base, respectively, store user personal information data, instructional resource related data, and all user behavior information tracked and recorded by the system. These data run through the interactive activities of the whole system and basically constitute the data sources required for personalized resource recommendation model.

## 4. Result Analysis and Discussion

The dance choreography course instructional management system developed and deployed in this study is in charge of centrally managing, organising, and presenting all instructional resources in the resource database. In addition, it assists in monitoring user activity, capturing the resulting user data, and providing thorough and significant user data for resource recommendation. In this paper, the resources are stored in multimedia server, database server, and file server, respectively, and whether to buffer each other's data resources is determined according to the actual needs. These resource servers not only provide Client/Server data request mode, but also provide Peer-to-Peer data sharing mode. The data access mode is determined according to the access request of the client. Considering the convenience and difficulty of development, the development and operation of the system are all carried out under Window. The system is mainly centered on educational grid laboratory, connected by Gigabit switching system, integrated with distributed laboratory, computer cluster laboratory, and NC-Linux laboratory, and provides interfaces for other user groups.

The article "Teaching of Dance Choreography Course Based on Multimedia Network Environment" was retracted in 2023. Reasons: unreliable results or conclusions; concerns about the data; concerns about the peer review; concerns about the citations.

User registration information collection mainly collects the demographic information of users, which is used for the analysis of user clustering and stored in the basic information table of users in the database. It mainly includes user information as shown in Table 1.

Through a browser, users log in to the system, access system resources, and use system features. Depending on their rights, users are classified as administrators, regular users, and guests. When users rate resources, the process of gathering user evaluation data is finished. The scores of users on certain resources are gathered and placed in the database's user rating table. The specific content of the user rating table is shown in Table 2.

The management node serves as the storage center and dispatch center of system information. Search the stored data, determine the location of users' on-demand movies, and cache and schedule videos.

In the improved algorithm of this paper, first of all, we need to find several similar concepts that are processed each time. These similar concepts that are processed once are required to have little difference in similarity, and the concepts with high correlation that we are looking for must be in other unprocessed high levels. Therefore, this paper introduces the difference of similarity to judge the similarity between layers. In this paper, based on the same user evaluation data, two similarity calculation methods are compared experimentally, and the average absolute error comparison chart of the following two algorithms is shown in Figure 3.

The experimental findings indicate that, using the same experimental data, the correlation similarity measurement method's recommendation quality is higher than the cosine similarity measurement method because the correlation similarity measurement method's error is obviously smaller than cosine similarity. Therefore, to identify the users who are the target users' neighbours, this study chooses the correlation similarity measuring approach.

This database mainly stores instructional resources in a certain form, including audio resources, video resources, document resources, and resource allocation list. Audio resources mainly refer to recording materials, lecture recording materials, etc. Video resources refer to all kinds of instructional resources in the form of images; the documents include courseware, electronic version of teaching notes, etc. The resource allocation list refers to the allocation of a certain resource among the resource servers, which is helpful to reposition the data request. In this paper, different similarity algorithms are used to cluster instructional resources, and the clustering results are shown in Figure 4.

The article "Teaching of Dance Choreography Course Based on Multimedia Network Environment" was retracted in 2023. Reasons: unreliable results or conclusions; concerns about the data; concerns about the peer review; concerns about the citations.

It can be seen that the similarity in this paper is much more accurate than the conceptual similarity calculated by simply using names and the traditional similarity calculation methods. Because the concept names generated from the database are not standardized, this paper adopts the concept similarity of concept names and attributes as the clustering standard. Experiment again, and the recall rates of different algorithms are shown in Figure 5. The precision of different algorithms is shown in Figure 6.

This system is extensible, transplantable and transparent, and it is applicable to the whole workflow of users. With the expansion of instructional resources, the continuous expansion of the system and the more frequent contact with the outside world, each major can unite with other systems or set up its own application service system, becoming another relatively independent node in the grid.  Table 3 shows the grid node table of this paper.

The generation of system load time series, in the prototype system, the system load should be calculated according to the usage of the main hardware resources in the system, and the system load should be determined mainly by referring to the usage of processor, memory, external storage, and network equipment. The system load is shown in Figure 7.

As can be seen from Figure 7, when the load balancing algorithm is turned off, the system load of the server increases rapidly with the increase of client visits. When the load balancing scheduling algorithm is used, although the load of the server will increase with the increase of access clients, it is generally better than that when the load balancing algorithm is turned off. In this paper, similar concepts are clustered on the basis of calculating the similarity of concepts. In this paper, the processing algorithm of clustering results and the relationship between concepts are used to integrate all ontologies into one ontology. Experimental results show that the recall and precision of the proposed algorithm can reach 95.71% and 96.84%, respectively. To some extent, it solves the problems of users' difficulty in finding needed instructional resources and low utilization rate of instructional resources.

## 5. Conclusions

A key factor in ensuring the smooth progression of dance choreography instructional courses is the incorporation of multimedia instructional methods. This practise has become an unavoidable trend in today's dance choreography education. In order to improve the teaching quality of choreography, relevant staff must deepen the reform of dance choreography teaching using information technology, learn more about multimedia theory and related technologies, and promptly apply them to dance teaching practise. This paper makes the argument that multimedia technology should be incorporated with dance art so that dance works can give audiences a deeper feeling and impression and promote the diversified development of dance art by outlining the characteristics of multimedia and its application advantages in choreography. In addition, it is suggested that in order to try something new in the teaching of dance choreography, the multimedia network classroom should utilise the diversity of instructional information, the interactivity of the instructional system, the real-time instructional feedback, and many other characteristics. Based on this, this paper makes an effort to build the instructional management system for a dance choreography course and plans and implements a workable plan for creating and integrating the course's instructional resources. A better flow scheduling technique and a cache replacement strategy are both suggested at the same time. According to experimental findings, the recall and precision of the suggested method can both approach 95.71% and 96.84%, respectively. This method addresses the issues that the hybrid method and multiontology method have with reusing current ontologies and adding new sources. It enhances the individuation and intelligence of the dance choreography course's instructional management system. Additionally, this approach partially addresses the issues of users' difficulties in locating necessary instructional materials and instructional resources' low use rate. We can investigate and research the standardised management and storage of educational resources in future work.

The article "Teaching of Dance Choreography Course Based on Multimedia Network Environment" was retracted in 2023. Reasons: unreliable results or conclusions; concerns about the data; concerns about the peer review; concerns about the citations.

## Figures and Tables

**Figure 1:** Architecture diagram of instructional management system of dance choreography course.

**Figure 2:** Structure diagram of instructional management system of dance choreography course.

**Figure 3:** Comparison of experimental errors of similarity measurement.

**Figure 4:** Clustering results of different similarity algorithms.

**Figure 5:** Recall rate of different algorithms.

**Figure 6:** Accuracy of different algorithms.

**Figure 7:** Load situation of the system.

**Table 1:** User information table.

Field name	Field type	Field description
PK_UserID	Sequence	User ID
FK_Gender	Byte	Gender
F_Birthdate	Date	Date of birth
F_SpareTime	Int	Free time
FK_FavPlace	Int	Prefer learning places
FK_FavTime	Int	Preferential learning time

**Table 2:** User rating table.

Field name	Field type	Field description
FK_UserID	Int	User ID
FK_KldID	Int	Instructional resource ID
F_Score	Int	Scoring value
F_ScoreDate	Date	Scoring time

**Table 3:** Grid node table.

Field	Type	Attribute	Field description
SID	Integer	Not null	Node ID
MAXRA TE	Integer	Null	Maximum performance index that a node can provide
DEMO	Varchar	Null	Program type description

## Data Availability

The data used to support the findings of this study are available from the corresponding author upon request.
